This article has been retracted.

# Evaluating the effects of air disinfectants in decontamination of COVID‐19 aerosols

**DOI:** 10.1002/hsr2.1042

**Published:** 2023-01-10

**Authors:** Soheil Dehghani, SeyedAhmad SeyedAlinaghi, Amirali Karimi, Fatemeh Afroughi, Shayan Abshenas, Kimia Azad, Marcarious M. Tantuoyir, Parsa Mohammadi, Seyed Mohammad Ghavam, Hengameh Mojdeganlou, Omid Dadras, Newsha Nazarian, Farzin Vahedi, Alireza Barzegary, Esmaeil Mehraeen

**Affiliations:** ^1^ School of medicine Tehran University of Medical Sciences Tehran Iran; ^2^ Iranian Research Center for HIV/AIDS, Iranian Institute for Reduction of High Risk Behaviors Tehran University of Medical Sciences Tehran Iran; ^3^ Pars Hospital Iran University of Medical Sciences Tehran Iran; ^4^ School of medicine Islamic Azad University Tehran Iran; ^5^ School of medicine Kashan University of Medical Sciences Kashan Iran; ^6^ Biomedical Engineering Unit University of Ghana Medical Center (UGMC) Accra Ghana; ^7^ Department of Pathology The Johns Hopkins University School of Medicine Baltimore Maryland USA; ^8^ Department of Global Public Health and Primary Care University of Bergen Bergen Norway; ^9^ Department of Health Information Technology Khalkhal University of Medical Sciences Khalkhal Iran

**Keywords:** aerosol, COVID‐19, decontamination, disinfectants, SARS‐CoV‐2

## Abstract

**Introduction:**

Airborne transmission is the most  crucial mode of COVID‐19 transmission. Therefore, disinfecting the severe acute respiratory syndrome coronavirus‐2 (SARS‐CoV‐2) aerosols float can have important implications in limiting COVID‐19 transmission. Herein, we aimed to review the studies that utilized various disinfectants to decontaminate and inactivate the SARS‐CoV‐2 aerosols.

**Methods:**

This study was a review that studied related articles published between December 1, 2019 and August 23, 2022. We searched the online databases of PubMed, Scopus, Web of Science, Cochrane, on August 23, 2021. The studies were downloaded into the EndNote software, duplicates were removed, and then the studies were screened based on the inclusion/exclusion criteria. The screening process involved two steps; first, the studies were screened based on their title and abstract and then their full texts. The included studies were used for the qualitative analysis.

**Results:**

From 664 retrieved records, only 31 met the inclusion criteria and were included in the final qualitative analysis. Various materials like Ozone, H_2_O_2_, alcohol, and TiO_2_ and methods like heating and using Ultraviolet were described in these studies to disinfect places contaminated by COVID‐19. It appeared that the efficacy of these disinfectants varies considerably depending on the situation, time, and ultimately their mode of application.

**Conclusion:**

Following reliable protocols in combination with the proper selection of disinfectant agents for each purpose would serve to achieve desired elimination of the SARS‐CoV‐2 transmission.

## 1 INTRODUCTION

Severe acute respiratory syndrome coronavirus‐2 (SARS‐CoV‐2) is a newly emerging virus that has been a critical global health concern for the past two years.^1^, ^2^, ^3^ In December 2019, the first cases of COVID‐19 were discovered in Wuhan, Hubei Province, China.^4^ Rapidly a pandemic was developed, which was announced by the World Health Organization on March 11, 2020.^5^ The virus is transmitted via airborne and direct contact with infected individuals (kissing and shaking hands) or surfaces.^6^

Airborne transmission has been divided into two distinct modes that do not require direct contact: (i) virus‐containing droplets and (ii) virus‐containing aerosols.^7^, ^8^ Although SARS‐CoV‐2 has been spreading through all the mentioned methods, it seems that airborne transmission may play the loading role in this rapidly spreading outbreak.^9^ For transmission of the virus through an airborne route, various factors like air conditioning, temperature, humidity, and the rate of infected people are essential.^10^

In general, aerosols are defined as liquid and solid particles, which are called ultrafine particles (≤5 μm), that can be produced by respiration, talking, mechanical ventilation, dental procedures, and other aerosol‐producing procedures.^11^, ^12^ Some in‐vitro studies have reported that SARS‐CoV‐2 could be viable for 3 h in an aerosol^13^ and could be retained in the ambient air for hours^14^ or could be transmitted > 2 m or 6 feet before falling on the ground due to gravity.^12^, ^15^ Infectious droplets produced by coughing or sneezing contain larger particles (>5 μm) and are believed to settle within <2 m or 6 feet away from the infected person who produces them.^16^, ^17^

Although there are some controversies about the role of aerosols in virus transmission,^13^, ^18^ there is now some strong evidence to consider aerosol spread as a major route in virus transmission.^7^, ^8^, ^19^ Studies have reported that asymptomatic carriers, who have no cough, sneeze, or direct contact could transmit the virus.^20^, ^21^, ^22^

Only a few previous studies focused on the need to curb transmission of SARS‐CoV‐2 by disinfecting the aerosols containing the virus.^8^, ^14^, ^23^ As far as we know, there are only two systematic reviews that address the inactivation of SARS‐CoV‐2 in aerosols.^24^, ^25^ As has been mentioned before, the most dominant form of this super spread of SARS‐CoV‐2 is airborne transmission. Although the inactivation of SARS‐CoV‐2 in aerosols to control its rapid transmission is crucial everywhere, the effectiveness and toxicity of disinfectants are also of concern.^26^, ^27^ Therefore, it is necessary to identify safe disinfectants that can be applied in public areas without evacuating people. Given the significance of SARS‐CoV‐2 spreading via aerosols,^8^, ^10^, ^28^ particularly in setting connected to healthcare, hospitals, dental units and aerosol‐creating conditions,^11^ it is critical to understand how to prevent it from spreading by disinfecting aerosols. Given the significance of SARS‐CoV‐2 spreading via aerosols,^8^, ^10^, ^28^ especially in crowded areas, hospitals, and aerosol‐creating conditions,^11^ it is critical to understand how to prevent it from spreading by disinfecting aerosols. Thus, we aimed to review the existing studies to find the best disinfectant method for eliminating the SARS‐CoV‐2 in aerosols to prevent COVID‐19 spread.

## 2 METHODS

### 2.1 Overview

This study was a review that studied related articles published between December 1, 2019 and August 23, 2022. This article was conducted in accordance with PRISMA (Preferred Reporting Items for Systematic Reviews and Meta‐Analyses) checklist (Supporting Information Material 1). We searched and retrieved the studies using keywords on online databases of PubMed, Scopus, Web of Science, and Cochrane, on August 23, 2022. The selected articles were imported into EndNote (Thomson Reuters), and duplicates were removed using both the “duplicate” function and manually. Four researchers screened the remaining records in a two‐phase process. First, Three independent researchers read the titles and abstracts of all studies to identify potentially relevant articles based on inclusion criteria. The full texts of selected studies were thoroughly reviewed afterward and checked against the inclusion criteria, and irrelevant records were excluded. Three independent reviewers screened the full texts of selected studies and extracted the necessary information. Any disagreements between these reviewers were addressed through discussion and consensus with other researchers.

### 2.2 Search strategy

We have decided to search a combination of keywords, including “Disinfectants,” “Aerosols,” “COVID‐19,” and their synonyms in the abovementioned databases. All relevant studies were included regardless of their publication stage. Search strategies are provided in Supporting Information Material 2 for each database. An example of search strategy for PubMed was as follows:

[COVID‐19] OR [SARS‐CoV‐2] OR [SARS‐CoV2] OR [2019‐nCoV] OR [Novel coronavirus].
[Aerosol] OR [Aerosols] OR [Virus‐containing aerosol] OR [Viral aerosol] OR [Airborne transmission] OR [Droplet] OR [Airborne particle] OR [N95 masks] OR [Bioaerosol] OR [Ambient air].
[Disinfection] OR [Disinfectant] OR [Disinfectants] OR [Decontamination] OR [Superior filtration] OR [Virusend] OR [TX‐10] OR [TiO2] OR [Alcohol] OR [Ozone].
[A] AND [B] AND [C].

### 2.3 Study selection

We included all original studies concerning the effects of various disinfecting methods on the SARS‐CoV‐2 aerosols that have been published in English. To improve the validity of our findings, the review included all the observational (prospective cohort, cross‐sectional, and case studies) and experimental (randomized controlled trials, pre−post design, quasi‐experimental) studies.

Exclusion criteria were as follows:

1. Nonoriginal studies, including reviews, systematic reviews, and meta‐analyses.
2. Case reports.
3. Abstract, conference abstracts, and studies with unavailable full‐texts.
4. Opinions, editorials, commentaries.

### 2.4 Data extraction

Three researchers thoroughly read and extract the data from included studies and organized them into a word table containing the author name, type of study, year of publication, disinfection agent, time of the viral reduction, amount of viral reduction, size of the particles, and summary of findings. Another independent researcher reviewed the extracted data and addressed any discrepancies and issues raised between other researchers.

## 3 RESULTS

A total of 664 articles were retrieved, of which 244 duplicates were removed, and 420 records remained for screening. Furthermore, 236 and 153 studies were excluded in the title/abstract and full‐text screening, respectively; and 31 articles were included in the final qualitative analysis (Figure 1).

**Figure 1:** PRISMA 2020 flow diagram for this review. PRISMA, Preferred Reporting Items for Systematic Reviews and Meta‐Analyses.

These studies reported various materials as well as methods that are used in viral as well as bacterial disinfection (Table 1). Disinfectants are used primarily to reduce the risk of viral transmission on contact surfaces and areas prone to aerosol contamination. Prominent disinfectants include Ultraviolet C (UVC), heat, ozone, electrostatic disinfector, H_2_O_2_, alcohol, and TiO_2_. These particular disinfectants are being used to reduce SARS‐CoV‐2 virus transmission. The efficacy of these disinfectants varies considerably depending on the situation, time, and ultimately their mode of application.

**Table 1:** Summary of the findings for all the included studies

ID	First Author	Country	Year of publication	Disinfection agent	Time of reduction	Reduction of viral infectivity	Size of particles	Summary of findings (e.g., efficacy of disinfectants, etc.)
1	Corrêa et al.^29^	Brazil	2021	UV–C		84%–97% in the hospital environments		This study was effective and safe by observing air disinfection standards using UV‐C technologies and can be repeated.
2	Feng et al.^30^	China	2021	UV + Filter in built environment		Close to 100%	two size ranges, one in the sub‐micron region (dp between 0.25 and 1.0 µm) and the other in super‐micron region (dp> 2.5 µm)	Size‐dependent filtration efficiency was close to 100%. The UV + filter is the most reliable and safe; while, consuming the highest energy. The proposed new design method for air purification systems could be an essential tool for controlling airborne diseases.
3	Feng et al.^31^	China	2021	Electrostatic disinfector (ESD)		100%		The well‐designed ESD disinfection efficiency (with a spatial charge density of 3.6 × 10−06 C/m^3^) can be up to 100%. Compared to HEPA, ESD can save 99% of energy which is consumed by HEPA without reducing disinfection efficiency.
4	Fiore et al.^32^	Italy	2021	H_2_O_2_	2 h			This method can be used not only for office paper‐based sensors but also for filtering paper‐based sensors, which increases the application of this easy method of mass correction.
5	Garcia de Abejo et al.^33^	Spain	2021	Low‐temperature‐steam–2%‐formaldehyde sterilization process				As a result, certain models of FFP2, FFP3, or N95 masks do not compromise their structure, fit, or filtering capacity in one or two disinfection cycles with 2% LTSF.
6	Hill et al.^34^	USA	2021	UV			1‐, 5‐, and 9‐mm (0.1 mm for the individual virion)	As the particle scale and UV absorption of the particle's material increase, Sp increases, and decreases.
7	John et al.^35^	USA	2021	N95 filtering face‐piece respirator with a peracetic acid room disinfection system	1 h and 16 min	~99%	~10^6^ colony‐forming units (CFU) of *G. stearothermophilus* spores and ~10^6^ plaque‐forming units (PFU) of bacteriophage MS2	PAA room HLDS are effective for the decontamination of N95 respirators in a short time
8	Kumar et al.^36^	India	2021	face masks following with different sterilization methods	30 and 60 min	100%	0.3–10 µm	When some measures, especially social distancing, are challenging to maintain the mask, it can provide more protection.
9	Lammers et al.^37^	USA	2021	blue surgical sterilization wrap for homemade respirator masks		95%	0.3 µm	The current claims, which show superior filtration results compared to medical‐grade N95 masks, are derived from a misinterpretation of industrial experiments.
10	Li et al.^38^	China	2021	an aggregation‐induced emission (AIE)‐active luminogen‐loaded nanofibrous membrane (TTVB@NM) sharing sunlight‐triggered photodynamic/photothermal anti‐pathogen functions are prepared using the electrospinning technique	5−10 min	>99%		A set of antimicrobial evaluations show that TTVB @ NM can effectively treat pathogenic aerosols containing bacteria (inhibition rate: >99%), fungi (~88%), and viruses (>99%) Turn off sunlight in just 10 min.
11	Mohan et al.^39^	India	2021	dioxide (ClO_2_)		Inactivates upto 99% of viruses	Remove virus and bacteriophages upto 0.001 m in size	Protein layer of enveloped and non‐enveloped viruses and RNA and DNA Inactivates by oxidizing.
				Ozone (O_3_)				
				Sodium hypochlorite (NaOCl) hydrogen peroxide (H_2_O_2_) peracetic acid (PAA)				
				Solar Nonionizing (UV)				
				Ionizing (gamma‐ray)				
				Slow sand and ceramic				
				Ultra‐filtration, Nano‐filtration, Reverse osmosis Membrane				
12	Parry et al.^40^	India	2021	62%–75% ethanol	3−4 times after a contact period of 1 min			62%–75% ethanol reduces infectivity of SARS‐CoV‐2 by 3 to 4 times after a contact period of 1 min. Sodium hypochlorite (NaClO) solution in a concentration of 0.1%–0.5% reduces the infectivity of the virus by 3 times after a contact period of 1 min. 2% glutaraldehyde and 0.5% H2O2 areequally efficient and reduce infectivity by 3 times after 1 min of contact time.
				(NaClO)				
				glutaraldehyde and 0.5% H_2_O_2_				
13	Percivalle et al.^41^	Italy	2021	zone at the three tested concentrations of 0.5, 1, and 2 ppm	40 min	99%		Ozone at the three tested concentrations of 0.5, 1, and 2 ppm significantly reduced the SARS‐CoV‐2 titerafter 40 min fumigation on all assessed surfaces, including FFP2 mask and surgical gown.
14	Schinkothe et al.^42^	Germany	2021	Dry fogging (aerosolized peroxyacetic acid and hydrogen peroxide)	48−52 h			Dry fogging is highly microbicidal, efficient, rapid, robust, and neutral. A low concentration of dispersed disinfectant entails high material compatibility. It is an ideal method for hospitals, public conveyances, and indoor areas.
15	Sharun et al.^43^	India	2021	Sunlight exposure (UVC)	9 min	Complete inactivation not achieved		Direct skin exposure promotes the production of vitamin D which can lower the risk of Respiratory Tract infections. The intensity of sunlight is highest near the equator; therefore they had lower fatality rates. Antimicrobial photodynamic therapy can be considered as an alternative therapeutic strategy.
16	Zucker et al.^44^	Israel	2021	Ozone (1000 ppm)	30 min.	99%		Ozone gas is an effective disinfectant for SARS‐CoV‐2 with high potential to overcome the low accessibility of commonly applied liquid disinfectants
17	Guo et al.^45^	China	2020	alcohol				Alcoholic disinfection for the nozzle and the surrounding air was effective in reducing germs in aerosols.
18	Gupta et al.^46^	India	2020	Negative Pressure Aerosol Containment Box				This type of innovation requires an hour to reduce the risk for HCW without compromising patient safety and comfort in an affordable manner.
19	Heo et al.^47^	Republic of Korea	2020	TiO2−CV		99.9%	1−2 mm	
				based VLA antimicrobial air filters				
20	Inagaki et al.^48^	Japan	2020	deepMN‐UV LED irradiation	10 s (for 99.9% reduction)	99.9%	150 μl	Virus‐infected cells irradiated for 60 s showed a morphology largely comparable to that of cloned cells.
21	Mijoska et al.^49^	Macedonia	2020	Ethyl alcohol (78%–95%), 2‐propanol (70%–100%), a combination of 45% 2‐propanol with 30% 1‐propanol, glutaraldehyde(0.5%−2.5%), formaldehyde (0.7%–1%), and Povidone‐iodine (0.23%–7.5%)	1 min	Eliminate virus infectivity by 4 log or more		Water and detergents in combination with common disinfectants should be used to clean operational and areas at high risk for the presence of the virus with 0.05% sodium hypochlorite diluted with water (1 g/L). For disinfection of smaller areas, 70% Ethanol can be used, which after 1 min of exposure showed a significant reduction in the vitality of coronaviruses.
22	Morawska et al.^50^	Australia	2020	germicidal ultraviolet (GUV, or UVGI—ultraviolet germicidal irradiation	5 min	With almost a 6 log reduction in 5 min	<2.5 µm	Under laboratory conditions, GUV has been shown to be effective against a suite of microorganisms including coronaviruses.
23	Raventos et al.^51^	Spain	2020	Hydroalcoholic aerosol (70% ethanol)	641 s	Removes all traces	*R* ^2^ = 0.9698	Air curtains equipped with sprayers thatdistribute HA droplets to surfaces, reduce the viral load. It represents an additional and manageable measure to rapidly and economically reduce the spread of the virus.
24	Ren et al.^52^	China	2020	Circulating wind ultraviolet air disinfectors				Circulating wind air disinfectors with high ultraviolet rays, kill the microorganisms and promote the flow of indoor air.
25	Rohit et al.^53^	India	2020	Ultraviolet radiation exposure, isopropyl alcohol dip, ethylene oxide, autoclave, plasma sterilization, dry heat sterilization	52‐min cycle	Over 95%	0.3−0.5 microns	Three N95 face masks of different make subjected to 6 decontamination methods. All sterilization retained over 95% efficiency, with autoclave showed a drop, and UV showed variations in the size of the particle after decontamination.
26	Tu et al.^54^	China	2020	in‐situ formed nickel oxide hydroxide(NiOOH) as anode catalyst and sodium carbonate(Na_2_CO_3_) as electrolyte	30 s	95%		Electrochemical disinfection approach to treat with the COVID‐19 via inactivating the SARS‐CoV‐2 virus in a water electrolysis process
					5 min	99.99%		
27	Vernez et al.^55^	Netherlands	2020	ultraviolet germicidal irradiation (UVGI) for FFR masks	600 mJ/cm^2^ (10 Cycles)	Particle penetration ratio < 5%−6%		Decontamination procedure for FFR masks is an attractive method for respirators in case of shortages during a SARS pandemic
28	Campos et al.^56^	USA	2020	Heat 75°C	30 min.	100%		Heating with temperatures of 75 − 85°C can efficiently inactivate the virus on melt‐blown polypropylene Fabriqueof N95 masks after 20−30 min without lowering filtration efficiency
				85°C	20 min.			
29	Widmer et al.^57^	Switzerland	2020	H_2_O_2_ Plasma		75%		H_2_O_2_ plasma sterilization for decontamination allows reprocessing filtering facepiece masks (FFP2), while they still meet the filtration efficiency
30	Wu et al.^58^	China	2020	Water Immersion Test	Meltblown:	79%, 99%		Three methods for disinfection of masks are successfully reliable ways for reusing masks
				75% Alcohol Solution	Nano:Meltblown:	50%, 99%		
				UV (long term)	Nano:Meltblown:Nano:	<100%		
						100%		
31	Xiang et al.^59^	China	2020	Dry Heat 70°C	1 h	100%	0.1−10 mm	Heating with temperatures of 70°C for 1 h can efficiently inactivate the H1N1virus on N95 masks without lowering filtration efficiency

The findings of the present review show that UVC is the most common method used in disinfecting objects mostly N95 masks, contaminated air, and other contact objects with the possibility of viral contamination. UVC efficacy ranges from 36.4% to 100%.^29^, ^30^, ^34^, ^48^, ^60^, ^61^ Efficacy variability is attributed to the mode of usage as reported by the studies.^30^, ^45^

Ozone as a physical disinfectant has very good efficacy in reducing viral transmissibility and infectivity.^62^ The most widely used substance or disinfection agent is alcohol with very high efficacy in reducing SARS‐COV‐2 viral infectivity and transmissibility.^40^, ^45^, ^49^, ^63^ Studies reported disinfection of face masks (N95) at 75−85°C for 20−30 min.^64^ This recycling of N95 masks also proved to be very effective with minimal disruption of the structure of the mask to deactivate the virus.^64^

## 4 DISCUSSION

The present pandemic has clearly affected almost every part of human life across the world. Although there are currently several vaccines available, their inability to confer full immunity coupled with a low vaccination uptake still drives the pandemic. It is therefore paramount to continue implementing other traditional ways of preventing and reducing infection with the virus such as using disinfectants and adhering to public health protocols since these are the most effective and primary strategies to reduce viral transmission. Inhalation of infectious particles dispersed in the air, direct deposition on mucosal membranes, and indirect contact via contaminated surfaces are all ways for the virus to spread. Aerosol‐mediated SARS‐CoV‐2 transmission has been well documented^57^, ^65^, ^66^; therefore, methods of disinfection that can reduce such transmission are critical to curb the pandemic and prevent future viral outbreaks. Based on the findings of the present review, the use of dry heat, UVC, chemical agents, titanium dioxide, ozone, electrostatic disinfector, and a novel disinfectant known as Virus end (TX‐10) are some of the aerosol and contact decontaminates that are being used in the current pandemic.

*Protection Approaches for Transmissions of SARS‐CoV‐2*

- Physical methods
  Ultraviolet radiations including UVC, UVA, UVB, visible light, and infrared radiation have germicidal activities. UVC as one of the germicidal agents is used in ultraviolet phototherapy. They are radiations with wavelengths ranging from 200 to 290 nm. Our analysis shows that UV‐C is the most common physical form of disinfecting objects mostly N95 masks, contaminated air, and other contact objects with the possibility of viral contamination including inactivating human CoVs and SARS‐CoV‐2 on environmental surfaces.^25^ This spells out the critical preventive role that it could play in the spread of the SARS‐CoV‐2 virus. Studies have postulated that nanofiber membrane in N95 masks and respirators maintained their filtration efficacy after being subjected to long‐term exposure under UV light or successive doses of 60 mg/cm^2^ after a short drying cycle (30 min, 70°C). It suggests that N95 masks and respirators can be disinfected and reused using ultraviolet germicidal irradiation, especially in resource‐limited conditions.^43^, ^55^, ^58^ However, further studies are needed to determine the number of successive reuse cycles that a single respirator or mask can undergo while maintaining its filtration efficacy.^53^
  Open‐air decontamination is also another way in which ultraviolet radiation can be employed. This method of application requires using high‐intensity UV rays (254 nm UV‐C). These circulating wind ultraviolet air disinfectors do not only kill pathogenic microorganisms in the air, but they also effectively improve the flow of indoor air by circulating wind; hence, they are very effective in eliminating SARS‐CoV‐2 aerosols.^25^, ^52^, ^67^, ^68^ Other reports indicate that SARS‐CoV‐2 viral load can be significantly reduced or even eliminated with as low as 10 s−3 min of UVC irradiation on contaminated surfaces of personal items.^61^ Aside from this method, upper‐room germicidal UV fixtures seem promising and effective in reducing and managing airborne transmissions. This could be applied in various viral respiratory outbreaks since it is an old technological measure known to be effective, safe, and economical.^33^, ^69^, ^70^
  There are, however, some disadvantages with this method. Human exposure to UVC may cause kerato conjunctivitis and erythema and requires protection of the skin and the eyes of people exposed to levels above recommended exposure limits. However, by enclosing the UVC sources or by irradiating in the absence of human activity, human exposure is eliminated.
  Another form of physical decontamination reported is the use of dry heat usually between 60°C and 85°C. With as low as 5 min to 1‐hour, dry heat applied to surgical face masks and N95 respirators showed efficient decontamination of SARS‐CoV‐2, human coronavirus NL63 (HCoV‐NL63), and chikungunya virus vaccine strain 181/25 (CHIKV‐181/25), without any reduction in the filtration ability as well as the structural composition of the masks and respirators. The efficiency of this particular method is very promising and nondestructive even at different relative humidity. It is regarded as the best method to sterilize N95 masks at 70°C−80°C. However, this method of decontamination can be repeated only 3 times on masks and respirators.^25^, ^36^, ^56^, ^59^, ^71^ Also, evidence demonstrates that autoclaving and dry heat at temperatures greater than 90°C cause physical degradation of melt‐blown fabric and consequently affects the filtration efficiency.^72^
- Chemical methods

Ozone (O_3_) is a physical disinfectant, a highly reactive gas that consists of three oxygen atoms. This particular gaseous disinfectant has been reported to be a very strong agent that can inactivate and consequently eliminate enveloped pseudoviruses including influenza A H1N1, MERS‐CoV, SARS‐CoV‐1, and SARS‐CoV‐2 even at minimal exposure in aerosols or fomites.^73^, ^74^ This method of disinfection has a positive correlation between surface hydrophilicity and disinfection. Its efficacy may depend on the type of surface it is being used on. Studies have reported that infected surfaces made of aluminum alloy are properly disinfected with ozone in comparison with surfaces like copper, nickel, and brass. There seems to be a gap in this regard and further studies may be needed to implement its usage on larger scales. Ozone is also effective in indoor locations with a good advantage over liquid disinfectants since it demonstrates similar decontamination in all surfaces including interior surfaces.^44^ Hence, using gaseous ozone as a sterilizing agent for high‐risk indoor rooms, PPEs, and crucial or difficult‐to‐reach surfaces, particularly in healthcare institutions, could help to limit the viral spread and maintain the safety of patients and healthcare professionals in the current pandemic as well as future outbreaks.^25^, ^41^ In reviewed works, low ozone exposures, just around 0.1–0.4 mg L‐1 min, achieve about 4 log10 of inactivation in aerosols, while exposures between 1 and 4 mg L‐1 min may be needed to guarantee an inactivation of 3–4 log10 in different fomites. Although further studies are required, ozone is an effective candidate to be used against SARS‐CoV‐2 or other viruses in surfaces and indoor locations. However, the uncertainties in front of a widespread use of ozone gas for virus inactivation are still significant.^74^

### 4.1 Titanium dioxide

Titanium dioxide (TiO₂) is an inorganic compound that has been reported by studies to possess multiantiviral effects. It is used to induce a photocatalytic reaction which proves to be an excellent disinfectant and can be used to tackle infectious diseases including SARS‐COV‐2.^47^ Furthermore, TiO_2_ is reported to be environmentally friendly, hence, does not have any substantial adverse effects on human health. However, it is time and medium dependent showing a faster disinfection rate for aerosols. Although this difference exists, the reduction in infectivity is similar.^75^ A novel disinfectant worth mentioning is Virusend (TX‐10). This antimicrobial agent is very effective in reducing SARS‐CoV‐2 virus transmission through indirect contact and aerosols. As a new method, it could be explored further for wide‐scale applications.^60^ Electrostatic disinfectors and elastomeric respirators have also been reported to have high disinfection and filtration efficiency, respectively. They both present highly efficient methods of terminating aerosol viral transmission.^54^, ^76^

### 4.2 Other chemical protection methods

As a chemical method, alcohol is the most widely used substance or disinfection agent with almost 100% efficacy in reducing SARS‐CoV‐2 viral infectivity and transmissibility. Many forms of chemical agents like ethanol, hydrogen peroxide, sodium hypochlorite, quaternary ammonium compounds, and phenolic compounds have been used successfully to inactivate the coronavirus on surfaces.^66^, ^68^ Plasma peroxide is also another chemical agent that is used in the decontamination of FFP2 respirators for recycling.^57^ A combinatorial chemical method formed from an aerosolized mixture of peroxyacetic acid and hydrogen peroxide (aPAA‐HP) demonstrates excellent disinfection ability against the SARS‐CoV‐2 virus. It is highly microbicidal, efficient, rapid, sturdy, eco‐friendly, and an effective form of airborne disinfection.^42^ The use of peracetic acid also proves to be very effective in decontaminating N95 respirators. This method is capable of disinfecting G. stearothermophilus spores as well as bacteriophage MS2. Therefore, this room disinfection system is effective in reducing SARS‐CoV‐2 viral transmission.^35^

The fact that all included studies are based on in vitro circumstances and that only a few thorough experiments attempt to replicate in vivo conditions is one of the major limitations of this systematic review. However, more investigation and evaluation are needed to determine the true efficacy of in vivo settings. The authors found it challenging to select papers that were both pertinent and of the highest caliber due to the large amount of research on COVID‐19. This was also one of the most notable study drawbacks.

## 5 CONCLUSION

To fully immune the population against SARS‐CoV‐2, we still need to continue using disinfectants, as the discovery of vaccines and antiviral drugs against COVID‐19 have not been as effective as expected in eliminating the incidence of new cases in the long term.

In this review we have gathered together the current knowledge of characteristics of available disinfection methods, such as UVC, heat, ozone, electrostatic disinfector, H_2_O_2_, alcohol, and TiO_2_, along with detailed instructions on for their appliance. Choosing the proper disinfectant that could serve our purpose is the first step; followed by adjusting the dosage to maximize the desired effect and reduce the side effects of the chemical or physical agents. A combination of proper timing, dosage, and type of disinfectants could ensure an effective decontamination process and safety of the user. Therefore, developing reliable protocols to use disinfectant agents is of great importance and future research should address that in each specific context.

## AUTHOR CONTRIBUTIONS

**Soheil Dehghani**: Writing – original draft. **SeyedAhmad SeyedAlinaghi**: Conceptualization; writing – review and editing. **Amirali Karimi**: Data curation; writing – original draft. **Fatemeh Afroughi**: Writing – original draft. **Shayan Abshenas**: Writing – original draft. **Kimia Azad**: Writing – original draft. **Marcarious M Tantuoyir**: Writing – review and editing. **Parsa Mohammadi**: Writing – original draft. **Seyed Mohammad Ghavam**: Writing – original draft. **Hengameh Mojdeganlou**: Writing – original draft. **Omid Dadras**: Writing – original draft; Writing – review and editing. **Newsha Nazarian**: Writing – original draft. **Farzin Vahedi**: Writing – original draft. **Alireza Barzegary**: Writing – original draft. **Esmaeil Mehraeen**: Conceptualization; writing – original draft; Writing – review and editing.

## CONFLICT OF INTEREST

The authors declare no conflict of interest.

## TRANSPARENCY STATEMENT

The lead author Esmaeil Mehraeen affirms that this manuscript is an honest, accurate, and transparent account of the study being reported; that no important aspects of the study have been omitted; and that any discrepancies from the study as planned (and, if relevant, registered) have been explained.

## Supporting information

Supporting information.

Supporting information.

## Data Availability

The authors stated that all information provided in this article could be share.
